The article "A Smart Healthcare Recommendation System for Multidisciplinary Diabetes Patients with Data Fusion Based on Deep Ensemble Learning" was published in 2021. Journal: Comput Intell Neurosci.

# A Smart Healthcare Recommendation System for Multidisciplinary Diabetes Patients with Data Fusion Based on Deep Ensemble Learning

**DOI:** 10.1155/2021/4243700

**Published:** 2021-09-17

**Authors:** Baha Ihnaini, M. A. Khan, Tahir Abbas Khan, Sagheer Abbas, Mohammad Sh. Daoud, Munir Ahmad, Muhammad Adnan Khan

**Affiliations:** ^1^Department of Computer Science, College of Science and Technology, Wenzhou-Kean University, Wenzhou 325060, China; ^2^Riphah School of Computing and Innovation, Faculty of Computing, Riphah International University, Lahore Campus, Lahore 54000, Pakistan; ^3^School of Computer Science, National College of Business Administration and Economics, Lahore 54660, Pakistan; ^4^College of Engineering, Al Ain University, Abu Dhabi 112612, UAE; ^5^Pattern Recognition and Machine Learning Lab, Department of Software, Gachon University, Seongnam 13557, Republic of Korea

## Abstract

The prediction of human diseases precisely is still an uphill battle task for better and timely treatment. A multidisciplinary diabetic disease is a life-threatening disease all over the world. It attacks different vital parts of the human body, like Neuropathy, Retinopathy, Nephropathy, and ultimately Heart. A smart healthcare recommendation system predicts and recommends the diabetic disease accurately using optimal machine learning models with the data fusion technique on healthcare datasets. Various machine learning models and methods have been proposed in the recent past to predict diabetes disease. Still, these systems cannot handle the massive number of multifeatures datasets on diabetes disease properly. A smart healthcare recommendation system is proposed for diabetes disease based on deep machine learning and data fusion perspectives. Using data fusion, we can eliminate the irrelevant burden of system computational capabilities and increase the proposed system's performance to predict and recommend this life-threatening disease more accurately. Finally, the ensemble machine learning model is trained for diabetes prediction. This intelligent recommendation system is evaluated based on a well-known diabetes dataset, and its performance is compared with the most recent developments from the literature. The proposed system achieved 99.6% accuracy, which is higher compared to the existing deep machine learning methods. Therefore, our proposed system is better for multidisciplinary diabetes disease prediction and recommendation. Our proposed system's improved disease diagnosis performance advocates for its employment in the automated diagnostic and recommendation systems for diabetic patients.

## 1. Introduction

A recent development in biotechnologies and high throughout computing progressively contribute to quick and affordable e-healthcare data collections and disease diagnosis. The efficiency and reliability are dependent on accurate model building from e-healthcare big data. One of many life-threatening diseases is diabetes disease (DD) [1–3].

The article "A Smart Healthcare Recommendation System for Multidisciplinary Diabetes Patients with Data Fusion Based on Deep Ensemble Learning" was published in 2021. Journal: Comput Intell Neurosci.

Diabetes disease arrests 422 million adults all over the world [4]. The death rate due to diabetes disease is 1.5 million, and 3.7 million deaths are due to diabetes and high blood pressure [4]. Diabetes disease is a multidisciplinary disease that arrests the human body's significant parts like the kidney, eyes, lungs, and heart. The diagnosis of this disease was done either manually by a medical practitioner or by any automatic device.

All of these types of measurements for diabetes disease have some benefits and some drawbacks. Any experienced medical expert cannot manually find the diabetes disease early due to some hidden side effects on the human body. With the intelligent recommendation system's help and application of deep machine learning (DML) and artificial intelligent methods, this disease can be predicted at the earlier stage [5–9] with a minimal error rate.

There are some healthcare automated systems for detection and recommendation of human diseases in recent researches. Myocardial infarction [10] is an acute disease for blood circulation in the heart. In this paper, deep CNN is applied for detection and to prevent humans from a heart attack. A computer-aided diagnosis (CAD) system [11] is used by applying the transfer learning technique for accurate and timely response to reduce the extensive calculation. In this paper, a CAD system works efficiently and accurately to detect and prevent heart attacks. Internet of Healthcare Things (IoHT) and Decentralization Interoperable Trust (DIT) [12] framework are a better healthcare system. In this paper, blockchain is used for data privacy and security. In this research, data is collected via IoHT at each point and transformed through blockchain for smooth and accurate healthcare data for better system accuracy.

Many ensemble learning models have been used in recent healthcare researches for better accuracy. For example, hepatocellular carcinoma [13] is a hazardous cancer disease in the human body. In this paper, an automated prediction system is developed using a stack learning approach for deep learning and examining healthcare data about this deadly disease. Stack learning is an ensemble learning technique. In this paper, evolutionary computational techniques are also used to examine the healthcare data about hepatocellular carcinoma disease. In cervical cancer [14] diagnosis, an ensemble machine learning approach is used. In this paper, two approaches are used for predicting disease on an images dataset.

The article "A Smart Healthcare Recommendation System for Multidisciplinary Diabetes Patients with Data Fusion Based on Deep Ensemble Learning" was published in 2021. Journal: Comput Intell Neurosci.

In mobile edge computing [15], an automated recommendation system is proposed for the joint computation of multiuser offloading and task caching. In this paper, Q-learning and Deep-Q-Network-based algorithms are proposed for this system. Multilevel vehicular edge cloud computing [16], secure federated learning for 5G [17], and augmented Coronavirus disease detection [18] used an advanced ensemble deep learning approach for better results.

For detection of COVID-19 disease, a deep learning approach is adopted with an augmented approach [18] and it achieved 100% accuracy. In industrial mobile edge computing [19], the deep ensemble learning approach is used for resource allocation and data security.

The importance of a smart healthcare recommendation system is increasing day by day for better and timely prediction. To minimize the risk of life-threatening human diseases, we need an efficient system for diagnosing and effectively recommending life-threatening diseases such as diabetes. Electronic health records (EHRs) play an essential role in smart healthcare recommendation systems for predicting life-threatening diseases, especially for multidisciplinary and life-threatening diabetes diseases. However, the data collected from sensors and EHRs are unstructured. To manage adequately such kinds of multisourced data for further examining is a challenging task.

Further, extracting the critical features and fusing them in a structured form is also a hectic and skills-demanding task. Therefore, this section is further divided into two parts: a wearable sensors-based diabetes prediction system and extracting information from EHRs textual data. Then, data fusion is essential for better results and accurate prediction of diabetes disease with DML.

Many recommendation systems for healthcare are already proposed in recent researches. The significant contribution of this research is to enrich the healthcare dataset for the best prediction of multidisciplinary diabetes disease. We have collected the patients' data through wearable sensors and EHRs in the textual record form of each patient. After collecting the records of each patient, essential data from both ends are fused to enrich the healthcare dataset. The Ensemble deep learning approach works accurately and produces better results in larger healthcare datasets. Finally, we have developed a better recommendation system by collecting patients' records and applying an ensemble machine learning approach for accurate and timely prediction and recommendation of multidisciplinary diabetes disease patients.

The article "A Smart Healthcare Recommendation System for Multidisciplinary Diabetes Patients with Data Fusion Based on Deep Ensemble Learning" was published in 2021. Journal: Comput Intell Neurosci.

The organization of the paper is as follows: Section 2 describes the most recent developments of diabetes disease detection and recommendation from the literature; Section 3 provides research methodology, data fusion, and proposed DML model; Section 4 presents the dataset selection, preprocessing, data fusion, and results and discussion; Section 5 describes the conclusion and future work; and the last section is devoted to references.

## 2. Related Work

Many researchers contributed to diagnosing diabetes disease. They have used machine learning (ML) classifier and artificial intelligence (AI) assistance for the prediction of diabetes disease. With the help of artificial intelligence, we can easily collect healthcare data. After collecting the big data from the healthcare center, we can easily predict human diseases, including multidisciplinary diabetes diseases.

In early detection of diabetes disease [20], the k-nearest neighbor (KNN) classifier model was used and the result was compared with that of the support vector machine (SVM) model achieving 85.6% accuracy. In this paper, the KNN machine learning classifier was used for predicting diabetes disease. The results comparison was made with another machine learning classifier called SVM to authenticate the work. For the detection of diabetes type II disease [21], the authors used a convolution neural network (CNN) and compared their work with the linear regression (LR) model and multilayer perceptron (MLP). In this paper, the neural network was used to diagnose diabetes type II disease. For results comparison, two machine learning classifiers were used for the authenticity of the work. An accuracy of 77.5% was achieved in the area under the curve (AUC). Analysis of early detection of diabetes disease with feature selection technique [22] was carried out using SVM classifier and their results were compared with random forest (RF), naïve Bayes (NB), decision tree (DT), and KNN classification models. The highest accuracy achieved with SVM was 77.73%. In this paper, the feature selection technique was adopted. With the help of the feature selection technique, we can reduce the system's computational capability and improve accuracy. Multiple machine learning models were applied for comparison and authenticity of results. Bloodless techniques for the prediction of diabetes disease are used with computational tools [23]. The accuracy achieved through this technique was 91.67%. In diabetic retinopathy detection [24], the deep (DNN) technique was adopted. The accuracy achieved via CNN was 74.4%. Detection of multiclass retinal disease [25] was done with with AI. The CNN classifier was used and it achieved 92% accuracy.

The article "A Smart Healthcare Recommendation System for Multidisciplinary Diabetes Patients with Data Fusion Based on Deep Ensemble Learning" was published in 2021. Journal: Comput Intell Neurosci.

A data-driven approach is used for predicting diabetes and cardiovascular diseases [26] with ML. This paper adopted an extreme gradient boost and compared it with the LR, SVM, RF, and weighted ensemble model. An accuracy of 95.7% was achieved in the area under the ROC curve. In type II diabetes disease prediction [27], an ensemble classification model was adopted. The accuracy achieved via this model was 82.2% in the AUC. A new methodology, smartphone-based diabetes detection [28], was presented. In this paper, image data was considered for diagnoses and further directions. A microcontroller-based agent [29] was used to measure the blood glucose level of patients. A sensor integrated therapy [30] for diabetes disease was used to monitor glucose levels in a diabetic patient. A self-recommendation smart app [31, 32] was used and trained on recorded health data like patients' daily physical activities and other important parameters related to diabetes.

The valuable information extraction from wireless sensor data and the patient's electronic medical record is also challenging for predicting multidisciplinary disease. To handle this challenge, different models have been presented for extracting the most valuable information from the healthcare textual data [33–35] for making a dataset for the prediction of diabetic disease. The textual dataset collected through EHR's was preprocessed and converted into a meaningful format as per smart healthcare recommendation system demands. The wireless sensor data of healthcare was also collected through wireless devices. After collecting data through a wireless communication device, data was preprocessed for removing noisy wireless data to make a rich and accurate healthcare dataset. In this way, we can easily apply machine learning algorithms for predicting multidisciplinary diabetes disease.

After collecting and converting meaningful data from textual data and fusing preprocessed wireless sensor data [36–38] for making a rich healthcare dataset of diabetes, Table 1 shows the comprehensive limitation of previously published approaches.

## 3. Smart Healthcare Recommendation System for Multidisciplinary Diabetes Patients

This section explains the overall structure of a smart healthcare recommendation system for multidisciplinary diabetes disease patients (SHRS-M3DP) in detail. The proposed approach is divided into distinct layers for an accurate description of each layer working. In the end, the ensemble DML structure is presented, which is further deployed in the whole SHRS-M3DP to predict and recommend diabetes disease in the patients. It should deliver a concise and accurate representation of the experimental results, explanation, and the conclusion of experiments that can be drawn.

The article "A Smart Healthcare Recommendation System for Multidisciplinary Diabetes Patients with Data Fusion Based on Deep Ensemble Learning" was published in 2021. Journal: Comput Intell Neurosci.

### 3.1. Smart Healthcare Recommendation System for Multidisciplinary Diabetes Patients

This part explains the overall structure of a smart healthcare recommendation system for multidisciplinary diabetes disease patients (SHRS-M3DP). Initially, the general structure of the proposed SHRS-M3DP is described. Then, a proposed system's structure is divided into distinct layers for an accurate description of each layer working. Finally, the ensemble deep learning model structure is presented, and it is further deployed in the whole SHRS-M3DP to predict and recommend diabetes disease in the patients.

The proposed structure of the SHRS-M3DP system is exhibited in Figure 1. It is divided into two main segments: (1) training phase and (2) validation phase. These phases are essential for the accurate prediction of multidisciplinary diabetes disease. These phases communicate via a cloud. The training phase comprises seven levels: (i) sensory layer, (ii) EHRs layer, (iii) raw feature layer-1, (iv) raw feature layer-2, (v) fused raw feature layer, (vi) preprocessing layer, and (vii) application layer. The sensory layer comprises input parameters, including age, family history, glucose, skin thickness, blood pressure (BP), pregnancies, insulin, and body mass index (BMI). The sensory layer's input values are collected and transferred to the database, raw feature layer-1, through the Internet of medical things (IoMT). Because wireless communication is applied, data collected from multiple feature nodes and stored in the database may be inaccurate. For that reason, we considered such kind of data as feature raw data. EHRs layer consists of lab reports, questions, observation, and the patient's medical history. All the data collected from the EHRs layer are reports and need some methodology to convert them into a structured format for further processing.

The Framingham risk factors (FRFs) methodology used in the smart healthcare monitoring system for heart disease prediction [39] is adopted to extract data from the EHRs, as shown in Figure 2, and stored in raw feature layer-2.

The data fusion approach is then applied for fusing the common features of both sensory data and EHRs to generate enhanced healthcare data on multidisciplinary diabetes disease.

These fused feature data are then stored in the fused feature layer for further processing to predict diabetes disease.

The following preprocessing layer plays a crucial role in the model. All deficiencies received through the sensory layer previously via wireless communication and EHRs layer are preprocessed in this phase. These missing values are managed by applying moving averaging and normalization methodology to mitigate noisy results. Subsequently, after preprocessing, the fused feature dataset is forwarded to the application layer. This layer is further divided into two sublayers: (i) prediction layer and (ii) performance layer. In the prediction layer, an ensemble DML model is applied to predict multidisciplinary diabetes disease.

The article "A Smart Healthcare Recommendation System for Multidisciplinary Diabetes Patients with Data Fusion Based on Deep Ensemble Learning" was published in 2021. Journal: Comput Intell Neurosci.

The ensemble deep learning combines several individual models to obtain better generalization performance of any predictive classification problem. The convergence process of the ensemble ML model is implemented in three ways: (1) max voting, (2) averaging, and (3) weighted average for classification.

The ensemble ML model used an advanced boosting technique for regularizing, limiting the overfitting issue, and producing better accuracy compared to other ML models. As a result, the response rate of the ensemble ML model is ten times faster compared to other ML models. In the ensemble ML model's boosting technique, the trained dataset is divided into multiple weak learners. The average error rate of one weak learner is updated in the next weak learner. Resultantly, the final strong learner was found to have a minimal error rate for prediction.

Ensemble deep machine learning classifier can be expressed as follows:

(1) $$\begin{array}{c} F\left(x\right)=\sum_{m}\alpha_{m}h_{m}\left(x\right), \end{array}$$

where *F*(*x*) is a strong learner of ensemble classifiers, *α*_*m*_ is weight calculated by considering the last iteration's error, and *h*_*m*_(*x*) is a weak learner

In this way, we can achieve maximum prediction accuracy. The operational flow of the advanced boosting ensemble DML model is shown in Figure 3 (Algorithm 1).

The results are then sent to the performance layer. In this layer, data received from the previous layer is calculated. The performance layer results are evaluated based on accuracy, precision, recall, F1, root mean square error (RMSE), and mean average error (MAE) achieved by the SHRS-M3DP model. After comparing results, “YES” indicates that our proposed SHRS-M3DP model successfully predicted diabetes disease, and “NO” means the prediction layer of the proposed SHRS-M3DP model will be modified till the learning criteria objectives are attained. After successfully training the proposed SHRS-M3DP model, the trained fused model moves to a cloud to further import and predict diabetes disease.

The validation phase comes in the last where trained fused SHRS-M3DP model is imported for prediction to authenticate whether the patient is affected with multidisciplinary diabetes disease based on the results.

The results are then sent to the next layer, called the performance layer. In this layer, the data received from the prediction layer is evaluated.

The article "A Smart Healthcare Recommendation System for Multidisciplinary Diabetes Patients with Data Fusion Based on Deep Ensemble Learning" was published in 2021. Journal: Comput Intell Neurosci.

The performance layer results are then evaluated based on accuracy, precision, recall, F1, root mean square error (RMSE), and mean average error (MAE) achieved by the SHRS-M3DP model. After comparing the results, “YES” indicates that our proposed SHRS-M3DP model successfully predicted diabetes disease, and “NO” means the prediction layer of the proposed SHRS-M3DP model will be updated until the learning criteria are achieved. After successfully training the proposed SHRS-M3DP model, the trained fused model moves to a cloud to further import and predict diabetes disease.

The last phase is the validation phase. In this phase, the trained fused SHRS-M3DP model is imported for recommendation to validate whether the patient is affected with multidisciplinary diabetes disease based on the results.

## 4. Experiments

The data collected from EHRs and sensors were discussed previously in the proposed SHRS-M3DP model. In addition, the fused feature database was also discussed in the last section. In this section, the proposed SHRS-M3DP model's performance is evaluated, and the results are discussed.

### 4.1. Dataset

The proposed SHRS-M3DP model is simulated with two different diabetes disease datasets: Hospital Frankfurt Germany diabetes dataset [42] and Pima Indians diabetes dataset. The Hospital Frankfurt Germany diabetes dataset consists of 2000 cases with eight features. The Pima Indians diabetes dataset consists of 768 patients with eight features. The fused features dataset for an experiment was made with the combination of features of both datasets. Both datasets' cases with some missing values are managed with proposed filtering, and normalization techniques were discussed earlier. The combined, fused dataset features are shown in Table 2. The fused features attributes, measuring units, and their ranges are also mentioned.

The fused features dataset consists of 2768 cases with eight features. A deep machine learning model cannot be utilized for the small dataset having nominal values. Therefore, all the nominal data is converted into numeric values for utilizing the ensemble deep learning model. Detailed features description of fused features is shown in Table 2.

### 4.2. Performance Evaluation

The experiment was carried out to indicate the proposed SHRS-M3DP model's performance for diagnosing diabetic disease. Initially, the data was collected from sensors, which were transferred through IoMT to the feature database. Similarly, the patients' data collected through lab reports, questions, observations, and medical history were converted from unstructured format to structure format for further preprocessing. After collecting the features from sensors and EHRs, both datasets' features were combined to make a rich health dataset for better prediction and recommendation of diabetes disease. Finally, the processing module analyzed the final combined, fused feature dataset for further processing.

The article "A Smart Healthcare Recommendation System for Multidisciplinary Diabetes Patients with Data Fusion Based on Deep Ensemble Learning" was published in 2021. Journal: Comput Intell Neurosci.

Furthermore, the Hospital Frankfurt Germany diabetes dataset and Pima Indians diabetes dataset were then utilized for training the diabetes disease prediction model. For evaluation purposes, the proposed ensemble deep learning model was compared with some other classifiers: SVM, LR, KNN, NB, RF, and DT. The proposed SHRS-M3DP model was used before and after the feature selection and performance was compared. The datasets were divided randomly into 80% and 20%, respectively, to train and test the models mentioned above in the proposed model.

### 4.3. Evaluation Metrics

Dissimilar evaluation metrics were used to conclude the model's overall efficiency, as shown in Table 3. With the accuracy metric's help, we can present the proposed deep learning model's overall predictive ability. In the confusion matrix, true positive (TP) and true negative (TN) determine the proposed classifier's capability to predict the absence and presence of diabetes disease. false negative (FN) and false positive (FP) identify the proposed model's total false prediction. Recall metric and precision metric calculate the sensitivity and success of the diabetes disease presented model individually.

The function measure (FM) metric is used for prediction accuracy. Root mean square error (RMSE) and mean absolute error (MAE) calculate the difference and absolute variations among the predicted and the actual values. The values of $y_{i},\hat{y_{i}}$ denote the total numbers of observations of the predicted values and the actual values, respectively.

### 4.4. Results

This section presents the results of the above-mentioned proposed model and a comparison with other classifiers, respectively. The complete details of all classifiers for diabetes prediction are divided into three parts: prediction of diabetes disease, Pima Indians diabetes dataset consisting of 768 cases with eight features, Hospital Frankfurt Germany diabetes dataset consisting of 2000 patients with eight features, and finally with fused features dataset having 2768 cases with eight features as shown in Table 2, respectively.

The proposed SHRS-M3DP ensemble deep learning model prediction accuracy with other baseline classifiers is shown in Figure 4. The comprehensive explanation of each classifier before data fusion and after data fusion is as follows:

- Learner regression classifier (LR): LR accuracy in dataset 1 is 74.6% for predicting diabetes disease with 786 cases. In dataset 2, LR performed better, with 77.7% accuracy with 2000 cases. Still, in the final data fusion dataset, the accuracy for LR's prediction of diabetes disease is decreased to 75.2% with 2786 cases.
- Naïve Bayes (NB): NB classifier's accuracy in dataset 1 is 72% for predicting diabetes disease with 786 cases. In dataset 2, NB performed better, with 76.5% accuracy with 2000 cases. Still, in the final data fusion dataset, the accuracy for LR's prediction of diabetes disease is decreased to 74% with 2786 cases.
- Random forest (RF): RF classifier's accuracy in dataset 1 is 74.8% for predicting diabetes disease with 786 cases. In dataset 2, RF also performed better, with 81.2% accuracy with 2000 cases. Still, in the final data fusion dataset, the accuracy of random forest's prediction of diabetes disease is decreased to 80.5% with 2786 cases.
- K-nearest neighbor (KNN): KNN classifier's accuracy in dataset 1 is 73.3% for predicting diabetes disease with 786 cases. In dataset 2, KNN also performed better, with 77.7% accuracy with 2000 cases. In the final data fusion dataset, the accuracy of predicting diabetes disease with KNN is also increased up to 80.8% with 2786 cases.
- Decision tree (DT): DT classifier's accuracy in dataset 1 is 74% for predicting diabetes disease with 786 cases. In dataset 2, DT performed better, with 83.7% accuracy with 2000 cases. In the final data fusion dataset, the accuracy of prediction of diabetes disease with DT is 84.3% with 2786 cases.
- Support vector machine (SVM): SVM classifier's accuracy in dataset 1 is 74.6% for predicting diabetes disease with 786 cases. In dataset 2, SVM performed better, with 84% accuracy with 2000 patients. In the final data fusion dataset, the accuracy for predicting diabetes disease with SVM is 84.3% with 2786 cases.

The article "A Smart Healthcare Recommendation System for Multidisciplinary Diabetes Patients with Data Fusion Based on Deep Ensemble Learning" was published in 2021. Journal: Comput Intell Neurosci.

The proposed ensemble deep machine learning model performed outstandingly as compared to all the baseline classifiers. The proposed ensemble DML classifier's accuracy in dataset 1 is 72.7% for predicting diabetes disease with 786 cases. However, it is low due to the small dataset. In dataset 2, ensemble ML performed better and achieved 91% accuracy with 2000 cases, higher than all other classifiers. In the final data fusion dataset, the accuracy of prediction of diabetes disease with the proposed ensemble ML model is 99.6%, having a minimal error rate.

The summary of performance metrics, accuracy, precision, recall, F1, root mean square error, and mean absolute error of selected datasets individually and data fusion datasets, is presented in Tables 4–6.

Different DML classifiers are compared with the proposed model by various evaluation metrics, as shown in Table 4. In this experiment, only Pima Indians diabetes dataset is considered, without feature selection technique. The performance of each metric on a given dataset is precisely shown in Table 4. The proposed model's overall performance is less compared to the other classifiers due to the small dataset and the absence of feature selection technique.

In Table 5, only the Hospital Frankfurt Germany diabetes dataset is considered, without feature selection technique. Different DML classifiers are compared with the proposed model by various evaluation metrics, as shown in Table 5.

The proposed model's overall performance is more outstanding compared to the other classifiers due to the large dataset, as shown in Figure 4. Therefore, our proposed deep machine learning model can achieve more accurate results concerning a higher dataset ratio. In this experiment, the proposed model achieved 91% accuracy, much higher compared to other DML classifiers. On the other hand, in this experiment, RMSE and MAE are also very low compared with different DML classifiers's RMSE and MAE.

In Table 6, both diabetes datasets are being considered with the data fusion technique. Different DML classifiers are compared with the proposed model by various evaluation metrics, as shown in Table 3. The performance of each metric on a given dataset is precisely shown in Table 6. The proposed model's overall performance is much higher compared to the other classifiers due to the fused technique by making a rich healthcare dataset. Our proposed model performed outstandingly due to the data fusion technique and produced extraordinary results. In this experiment, the proposed model achieved 99.64% accuracy, much higher compared to other DML classifiers. In this experiment, RMSE is 0%, and MAE is only 0.06%. As shown in Table 6, all other classifiers produce results less than 85%.

Our proposed model accurately performed well with the help of data fusion technique. Our proposed ensemble DML model has achieved higher accuracy compared to other studies done in the recent past. The details of recent studies on diabetes with their authors are also summarized and shown in Table 7. The significant contribution for higher accuracy in our model is due to data fusion. In this way, we have made a rich healthcare dataset for the prediction of multidisciplinary diabetes disease. In this way, we have achieved higher accuracy compared to other studies, which is 99.6%.

## 5. Conclusion

The prediction of human diseases, particularly multidisciplinary diabetes, is challenging for better and timely treatment. A multidisciplinary diabetes illness is a life-threatening disease worldwide which attacks major essential human body parts. A proposed SHRS-M3DP model is presented to predict and recommend multidisciplinary diabetes disease in the patients quickly and efficiently. The ensemble deep ML model and data fusion technique are used for fast response and better accuracy rate. The proposed model efficiently predicted and recommended whether the patient is a victim of multidisciplinary diabetes disease or not. The proposed SHRS-M3DP model can also identify the effect of human body parts: Neuropathy, Retinopathy, Nephropathy, or Heart. The proposed SHRS-M3DP model simulation is made by using Python language. Finally, the study of this research concluded that the proposed SHRS-M3DP model's overall performance is 99.6%, which is outstanding compared to previously published approaches.

The article "A Smart Healthcare Recommendation System for Multidisciplinary Diabetes Patients with Data Fusion Based on Deep Ensemble Learning" was published in 2021. Journal: Comput Intell Neurosci.

### 5.1. Contribution

Many recommendation systems for healthcare have already been proposed in recent researches. The significant contribution of this research is to enrich the healthcare dataset for the best prediction of multidisciplinary diabetes disease. We have collected the patients' data through wearable sensors and EHRs in the textual record form of each patient. After collecting the records of each patient, essential data from both ends are fused to enrich the healthcare dataset. The ensemble deep learning approach works accurately and produces better results in larger healthcare datasets. Finally, we have developed a better recommendation system by collecting patients' records and applying an ensemble machine learning approach for accurate and timely prediction and recommendation for multidisciplinary diabetes disease patients. The overall performance of our recommendation system is 99.6%. In this way, future academic research and practices will be helpful for new researchers in this medical field, especially for automated prediction and recommendation systems for human diseases.

### 5.2. Future Work

The proposed SHRS-M3DP recommendation system achieved overall good performance. However, there is still a need to work for a better generalized efficient prediction and recommendation system for all human diseases. The complexity of the deep ensemble algorithm will also be considered in the near future for accurate and quick results of this algorithm.

## Figures and Tables

**Figure 1:** Proposed SHRS-M3DP model.

**Figure 2:** EHRs record conversion flow chart [40].

**Figure 3:** Flow chart of ensemble ML algorithm [41].

**Figure 4:** Accuracy of models before and after data fusion.

**Algorithm 1:** Algorithm 1 Ensemble ML-based diabetes prediction.

**Table 1:** Summary of existing literature reviews.

Paper	Classification methodology adopted	Limitations	Advantages
[12]	ML	1. Single dataset 2. No data fusion 3. Only structured data	Only the optimal feature selection technique was adopted
[13]	ML and AI	1. Single dataset 2. No data fusion 3. Only DR image data	The bloodless technique was adopted
[18]	DML and generalized linear model	1. Single EHRs dataset 2. No data fusion	1. Electronic health record 2. Data fusion 3. Feature selection
[19]	AI	1. Single dataset 2. No data fusion 3.Only DR image data	1. Automated software 2. Smartphone-based DR and sight-threatening detection
[20]	AI and ML	1. Single dataset 2. No data fusion	Incorporating wearable devices and IoT to collect and manage big data
[29]	Supervised ML	1. Single dataset 2. No data fusion	1. Combine structured and unstructured data 2. Feature selection

The article "A Smart Healthcare Recommendation System for Multidisciplinary Diabetes Patients with Data Fusion Based on Deep Ensemble Learning" was published in 2021. Journal: Comput Intell Neurosci.

**Table 2:** Feature information about the diabetes disease.

Sr. no.	Attribute	Unit	Ranges
1	Age	Year	01–120
2	Family history	Yes (1), no (0)	0, 1
3	Glucose	mg/Dl	37–380
4	Skin thickness	Mm	0–210
5	Blood pressure (BP)	mm Hg	90–190
6	Pregnancies	Number (0–9)	0–8
7	Insulin	uU/ml	0–764
8	BMI	Kg/m^2^	14–80.6
9	Diagnosis result	Positive (1), negative (0)	1, 1

**Table 3:** Performance metrics.

Name of metric	Description	Equation #
Accuracy (Acc)	(TP +TN)/( TP+TN +FP + FN )	(a)
Precision (Pre)	TP /(TP+FP)	(b)
Recall (Rec)	TP /(TP+FN)	(c)
F1-measure (FM)	((2 ^*∗*^Pre ^*∗*^Rec)/(Pre+Rec))	(d)
RMSE	$\sqrt{1/N}\sum_{i=1}^{N}{\left(y_{i}-{\hat{y}}_{i}\right)}^{2}$	(e)
MAE	$\sqrt{1/N}\sum_{i=1}^{n}{\left|y_{i}-{\hat{y}}_{i}\right|}^{2}$	(f)

**Table 4:** Comparison results of the proposed model with other classifiers before data fusion on the Pima Indians diabetes dataset.

Classifier model	Acc (%)	Pre (%)	Rec (%)	FM (%)	RMSE	MAE
Logistic regression	74.68	0.68	0.52	0.59	0.25	0.50
Naïve Bayes	72.08	0.62	0.52	0.57	0.28	0.53
Random forest	74.68	0.69	0.50	0.58	0.25	0.50
K-nearest neighbors	73.38	0.67	0.48	0.56	0.27	0.52
Decision tree	74.03	0.63	0.63	0.63	0.26	0.51
Support vector machine	74.68	0.70	0.48	0.57	0.25	0.50
^*∗*^ **Proposed model**	72.73	0.63	0.56	0.59	0.27	0.52

**Table 5:** Comparison results of the proposed model with other classifiers before data fusion on the Hospital Frankfurt Germany diabetes dataset.

Classifier model	Acc (%)	Pre (%)	Rec (%)	FM (%)	RMSE	MAE
Logistic regression	77.75	0.71	0.58	0.64	0.22	0.47
Naïve Bayes	76.50	0.67	0.61	0.64	0.24	0.48
Random forest	81.25	0.75	0.69	0.71	0.19	0.43
K-nearest neighbors	77.75	0.71	0.59	0.65	0.22	0.47
Decision tree	83.75	0.73	0.83	0.78	0.16	0.40
Support vector machine	84.00	0.79	0.73	0.76	0.16	0.40
^*∗*^ **Proposed model**	91.00	0.89	0.84	0.86	0.09	0.30

The article "A Smart Healthcare Recommendation System for Multidisciplinary Diabetes Patients with Data Fusion Based on Deep Ensemble Learning" was published in 2021. Journal: Comput Intell Neurosci.

**Table 6:** Comparison results of the proposed model with other classifiers after data fusion on a fused dataset.

Classifier model	Acc (%)	Pre (%)	Rec (%)	FM (%)	RMSE	MAE
Logistic regression	75.27	0.67	0.55	0.61	0.25	0.50
Naïve Bayes	74.01	0.64	0.55	0.59	0.26	0.51
Random forest	80.51	0.75	0.65	0.70	0.19	0.44
K-nearest neighbors	80.87	0.77	0.63	0.70	0.19	0.44
Decision tree	84.30	0.77	0.78	0.77	0.16	0.40
Support vector machine	84.30	0.81	0.71	0.76	0.16	0.40
^*∗*^ **Proposed model**	99.64	1.00	0.99	0.99	0.00	0.06

**Table 7:** Summary of comparison using diabetes datasets with existing methods.

Sr. no.	Author/year	Fusion method	Classifier/compared with classifier	Overall accuracy
1	Mohebbi et al. [10]/2017	—	CNN/LR, MLP	77.5%
2	Sneha and Gangil [11]/2019	Yes/—	SVM/RF, NB, KNN, DT	77.7%
3	Nguyen et al. [16]/2019	—	Ensemble ML/—	82.2%
4	Aminah and saputro [9]/2019	—	KNN/SVM	85.6%
5	Sah and sarma [12]/2018	—	AI	91.6%
6	Dinh et al. [15]/2019	—	XGB/LR, SVM, RF, weight ensemble model	95.7%
7	**Proposed method**	Yes/yes	Ensemble deep machine learning classifier/LR, NB, DT, KNN, RF, SVM	99.6%

## Data Availability

The data used in this paper can be requested from the corresponding author.
